The article "Analysis of Network Resources Integration of Political Thought Courses in Institution of Higher Learning Based on Collaborative Education Environment" was retracted in 2023. Reasons: unreliable results or conclusions; concerns about the data; concerns about the results or conclusions; concerns about the peer review.

# Analysis of Network Resources Integration of Political Thought Courses in Institution of Higher Learning Based on Collaborative Education Environment

**DOI:** 10.1155/2022/7989779

**Published:** 2022-08-31

**Authors:** Fengfeng Li

**Affiliations:** Jiangxi University of Finance and Economics,College of Marxism, Nanchang 330013, Jiangxi, China

## Abstract

The importance of political thought courses in higher education institutions is directly related to the caliber and extent of staff development. This essay carefully examines and discusses the integration of network resources for political thought courses in higher education institutions from the standpoint of collaborative education. This article analyses the current state of the integration of network resources into higher education institutions' political thought curricula. The general DM process and DM-related technologies are studied concurrently. The mining model based on the study of political thought course is chosen in conjunction with this course. Additionally, a teaching resource integration method based on the idea of collaborative learning is developed, including the development of an Arduino device identification program based on NN and an Arduino device learning resource base. In accordance with the design of the network resource integration method used in the political thought course, the article evaluates the model's performance in a number of different areas. The proposed algorithm's accuracy is 95.11 percent, according to experiments. The recall rate of this algorithm can also go as high as 93.94 percent. In order to further reform teaching and raise the standard of learning, this study can offer students learning direction.

## 1. Introduction

Political thought education serves to cultivate all-around development. Under the new historical conditions, cultivating high-quality socialist builders and successors is inseparable from cultivating their ideological and moral quality and scientific and cultural level. As a member of political thought theory course in an institution of higher learning, its development urgently needs the effective support of network teaching resources [1]. Network resources refer to the information content of resources in the Internet space. In the university environment where information-based teaching has been applied, almost every discipline will save the corresponding teaching resources to provide professional teaching for students, and so does political thought education [2]. Network teaching resources are divided into broad and narrow categories. Broadly speaking, network teaching resources refer to all kinds of related hardware resources and software resources. In a narrow sense, online teaching resources mainly refer to teaching resources transmitted in the form of a network, usually including video, multimedia resources, testing resources, etc. Network teaching resources usually exist in the form of a network teaching resource bank. With the continuous updating of the idea of running a school, the call for mutual benefit and resource sharing among institutions of higher learning is getting higher and higher, which further promotes the integrated development of online teaching resources in institutions of higher learning. The effectiveness of network teaching is affected by a number of important factors, including the quality of network course construction during the implementation process [3]. This course's application can, to some extent, reflect the course's richness and perfection in terms of resource allocation types and quantity. Fully grasp the necessity of using network resources in classroom instruction for political thought courses in higher education institutions, and deeply analyze the current situation and issues with using network resources; Next, actively explore how to integrate the network resources, while also making rational use of the network resources in classroom instruction, which is a crucial topic at this time for political thought teachers in higher education institutions [4]. Determining the best way to incorporate network teaching resources into a course on political thought theory is therefore unquestionably of great practical importance.

The article "Analysis of Network Resources Integration of Political Thought Courses in Institution of Higher Learning Based on Collaborative Education Environment" was retracted in 2023. Reasons: unreliable results or conclusions; concerns about the data; concerns about the results or conclusions; concerns about the peer review.

From the perspective of classroom teaching of political thought courses in institutions of higher learning, network resources are all information resources that can be used in classroom teaching of political thought courses in institutions of higher learning through the Internet. It has a huge capacity and rapid update; rich in content and diverse in forms; high sharing degree and easy access; complex, disorderly, and diverse characteristics [5]. At present, most teachers of political thought courses in institutions of higher learning realize the importance of network resources and make use of them in classroom teaching. Although many institutions of higher learning have implemented online teaching of political thought theory courses, the development of online teaching of political thought courses is restricted by the unsatisfactory construction of online teaching resources [6]. Massive data and lack of information are common embarrassments faced by all network teaching information systems after large data concentration. At present, most of the databases implemented by the network teaching platform can only realize low-level functions such as data input, query, and statistics, but cannot find all kinds of useful information in the data [7]. In order to better realize the educational goal of political thought education in institutions of higher learning, it is beneficial to integrate the concept of collaborative education into all facets of students' political thought education. By establishing and perfecting a cooperative education mechanism for college students' political thought education, different educational resources can be integrated, their advantages can be complemented, and the educational impact of political thought education can be increased [8]. The integration of network resources for political thought courses in institutions of higher learning is studied and analyzed in this article using DM (data mining) technology from the standpoint of collaborative education. The article's innovations are listed as follows:

1. This article, which examines the classroom instruction of political thought courses in higher education institutions, the research on network teaching resources integration and the research on network teaching of political thought theory courses in higher education institutions are organically combined. The advantages of integration are fully exploited in order to enhance the quality of political thought course instruction.
2. This article puts forward the importance of the integration of network teaching resources of political thought theory courses in institutions of higher learning. And through the integration of educational resources, formulate feasible collaborative education mechanisms to enhance the effectiveness of political thought education in institutions of higher learning.

The article "Analysis of Network Resources Integration of Political Thought Courses in Institution of Higher Learning Based on Collaborative Education Environment" was retracted in 2023. Reasons: unreliable results or conclusions; concerns about the data; concerns about the results or conclusions; concerns about the peer review.

## 2. Related Work

At present, many teachers of political thought courses in institutions of higher learning do not know enough about the necessity of using network resources in classroom teaching, and there are various problems with using network resources. Therefore, it is obvious that it is of great practical significance to explore how to integrate the network resources and make rational use of them in the classroom teaching of political thought courses in institutions of higher learning. Many scholars have studied it.

The discourse dilemma in the classroom teaching of political thought courses in higher education institutions was brought up by Nakayama et al. Political thought teachers' discourses are rather dated, lack vividness, the theory is disconnected from reality, and it is not persuasive or appealing [9]. The integrated use of AI in education was investigated by Cuevas et al. [10]. According to the study, AI technology is widely used in education and has the ability to personalize and interactively implement the teaching process while presenting educational content in a multimedia and networked manner. Significant changes have been brought about by educational evaluation. Dascalu and others contend that the organic unity of cognition, aptitude, and consciousness is one of the teaching goals of political thought courses. At the same time, the main method and foundation of moral education in schools is the teaching of political thought courses [11]. Zhang noted that many teachers are used to a self-centered and self-respecting teaching style, and that political thought teachers in institutions of higher learning use monotonous teaching methods. The effectiveness of political thought courses in institutions of higher learning is significantly impacted by the lack of exchanges, discussions, and interactive participation in classroom teaching [12]. According to Xu et al. artificial intelligence (AI) technology can significantly aid in the creation and integration of educational resources. Although using AI technology has a relatively high threshold, using teaching resources that are based on AI technology lowers that threshold significantly for students [13]. According to Lin, improving the collaborative educational construction of political thought courses in higher education institutions is a crucial step toward addressing the shortcomings of these courses, enhancing the effectiveness of instruction, and raising the standard of instruction [14]. Huang emphasized that educators must think about more than just how to incorporate interactive networks into the classroom because these networks cannot, on their own, have any educational impact. The interactive network will only have a significant educational impact when it is extremely closely related to the educational objectives of the school and the students' learning process [15]. According to the characteristics of modern educational technology and political thought courses, Kardan et al. specifically listed the application of several teaching modes in the integration of modern educational technology and political thought teaching, combining theory with practice to promote the smooth progress of the integration [16]. Hoxby pointed out that the current integration of teaching resources in political thought theory courses has the phenomenon of blind accumulation of resources, complex resource structure, and aging resource content. Under the guidance of political thought education theory, the cultivation of college students' moral quality, knowledge quality, and ability quality have become the target orientation of the integration of online teaching resources for political thought theory courses [17]. Kelly explored a new model of collaborative education, combining the Internet, mental health education, innovation and entrepreneurship education, and political thought work, and focused on exploring a collaborative education model for college students' political thought education that adapts to the specific conditions of institutions of higher learning [18]. Zobel et al. made a preliminary discussion on the contradiction between teaching and learning in online teaching, the contradiction between teacher-led and student-centered, modern educational technology and traditional teaching methods, and how to integrate network resources, technology, and political thought courses [19].

The article "Analysis of Network Resources Integration of Political Thought Courses in Institution of Higher Learning Based on Collaborative Education Environment" was retracted in 2023. Reasons: unreliable results or conclusions; concerns about the data; concerns about the results or conclusions; concerns about the peer review.

Currently, there is a slight lack of theoretical research on the integration and use of network resources in the classroom teaching of political thought courses in institutions of higher learning, and this practice is still largely unstructured, unconscious, and unstandardized. The integration of network resources for political thought courses in higher education institutions is studied and analyzed in this article using DM technology from the standpoint of collaborative education. The design of the Arduino device identification program based on NN (neural network) [20, 21] and the creation of the Arduino device learning resource database are part of the teaching resources integration method that is based on the idea of collaborative education. We should integrate educational resources and create workable cooperative education mechanisms in order to increase the effectiveness of political thought education in institutions of higher learning.

## 3. Methodology

### 3.1. Cooperative Education Mechanism of Political Thought Education

As the main channel of political thought education in an institution of higher learning, political thought courses in institutions of higher learning shoulder the important responsibility and mission of educating people. However, at present, the classroom teaching situation of political thought courses in institutions of higher learning is not optimistic, and some problems still exist, such as backward teaching ideas, outdated teaching methods, separation of theory from practice of the times, and weak effectiveness, which seriously affect the full play of its main channel. Collaborative education is an important concept that meets the requirements of the development of higher education. Applying collaborative education to the whole process of political thought education mechanism construction in institutions of higher learning is not only a response to the reform of higher education, but also an important driving force to improve the quality of talent cultivation in institutions of higher learning. It is of great theoretical significance and practical value to strengthen the construction of network teaching resources of political thought theory courses in institutions of higher learning and to carry out research on solutions. At present, in the process of collaborative education in online teaching, teachers and students are faced with the challenges of negative factors such as lagging concepts and insufficient skills, which greatly affect the promotion of collaborative education in the online teaching of political thought courses in institutions of higher learning. As a new concept and mode of political thought education, the cooperative education mechanism of political thought education for college students has the following characteristics:

① Systematization
② Interaction
③ Dynamic
④ Constituent elements

The primary method of educating college students about political thought is through classroom instruction in institutions of higher learning. We must fully exploit the guiding role that classroom instruction of political thought courses plays in institutions of higher learning if we are to further strengthen and enhance the political thought education provided to college students. The challenge for teachers in the environment of political thought education in institutions of higher learning is always how to effectively improve the comprehensive teaching effect of theoretical courses. Theoretical courses for students typically involve a lot of theoretical material, and they are limited to memorizing and comprehending the knowledge points provided by teachers. The current generation college students' learning needs are not being met by the learning process, which is too passive. Political thought education is a discipline with strong theoretical and practical characteristics. A deeper study of it is inseparable from a deep understanding and grasp of its related theoretical knowledge, and so is the research on the cooperative education mechanism of political thought education for college students. Strengthening the collaborative education construction of political thought course network teaching in institutions of higher learning is an important way to make up for the shortcomings of political thought course teaching in institutions of higher learning, improve the teaching effect, and also an important measure to improve the teaching quality. A successful political thought teaching course must, among other things, reflect cutting-edge educational concepts, reflect the standards of quality education, give full play to students' primary roles and cultivate students' autonomy in learning, adhere to educational laws, and accomplish specific educational objectives. The vast potential of the network enables communication between individuals from various regions, mobilizes people from various roles and responsibilities to work together, and connects thousands of computers. However, given the state of online education today, it is common to encounter slow content updates and out-of-date knowledge bases, which can have a negative impact on both teachers' and students' productivity. The development of network teaching resources is also insufficient. Finally, the network teaching platform's construction is flawed.

The article "Analysis of Network Resources Integration of Political Thought Courses in Institution of Higher Learning Based on Collaborative Education Environment" was retracted in 2023. Reasons: unreliable results or conclusions; concerns about the data; concerns about the results or conclusions; concerns about the peer review.

Establishing and perfecting the cooperative education mechanism of college students' political thought education can integrate various educational resources, complement each other's advantages and enhance the educational effect of political thought education. The complex and diverse ideas on the Internet aggravate the confusion and perplexity of college students, and erode their ideological and moral concepts. At the same time, the network also provides conditions for the innovation of classroom teaching of political thought courses in institutions of higher learning. Network environment resources refer to all kinds of equipment that ensure the normal operation of the network. Whether the network environment resources are good or not will affect the efficiency of teachers and students in using network resources, and will further affect their enthusiasm in using network resources [22]. The nature and task of the political thought discipline determine that we must always adhere to the principle of integrating theory with practice in the teaching of political thought courses, and we must always emphasize the leading role of teachers to implement the principle of combining indoctrination with persuasion. While the Internet has brought great impact to the classroom teaching of political thought courses in institutions of higher learning, it has also brought unprecedented opportunities. Network information resources refer to all kinds of information collections in the form of knowledge, data, information, news, and so on. There are two kinds of network resources in political thought courses: ① campus network and ② internet resources. The first is the intranet resources edited by the teacher team, which can only be spread in the campus network environment. The second is the free information resources that schools cannot control, and even the state cannot accurately control the content.

### 3.2. Utilization of Network Resources of Political Thought Courses in Institution of Higher Learning

Political thought education cannot keep students in fixed thinking, but it should expose them to various thoughts and cultures of various countries, and finally guide them to identify with socialist thoughts, so that their political thoughts can be correct and firm. And network resources can just enhance students' horizons, so that students can get more comparative information in their spare time. Therefore, network resources can also provide new ideas for political thought education. At present, most teachers of political thought courses in institutions of higher learning realize the importance of network resources and make use of them in classroom teaching. On the whole, teachers of political thought courses in institutions of higher learning are more active in using network resources, but the results are not good and the efficiency is not high. Many teachers focus on the use of network resources, neglect the selection and processing of network information resources, and neglect the organic combination of the use of network resources and traditional teaching methods. For teachers, the original way of preaching cannot meet the needs of online teaching. Students can use the Internet to freely acquire all kinds of knowledge they want, and teachers should change the teaching idea of monopolizing classroom speech and constantly update the teaching idea. In the process of constantly establishing and perfecting the mechanism, we should focus on the “education,” integrate high-quality resources within, between, and outside universities, and incorporate all kinds of education elements into the cooperative education mechanism system of political thought education for college students, so as to promote the cooperation and interaction among all elements. Classroom teaching is the main channel for talent cultivation, and it is also an important way for students to survive and develop. Teachers' leading role in teaching cannot be weakened, students' dominant position cannot be ignored, and the standardization and demonstration of textbooks cannot be changed. Otherwise, a good audio-visual operator, not a good teacher, will lose the real purpose of educational reform, and even fail to complete the teaching plan and teaching objectives. The classification of network teaching resources of political thought theory courses in institutions of higher learning is shown in Figure 1.

The article "Analysis of Network Resources Integration of Political Thought Courses in Institution of Higher Learning Based on Collaborative Education Environment" was retracted in 2023. Reasons: unreliable results or conclusions; concerns about the data; concerns about the results or conclusions; concerns about the peer review.

In order to improve the effect of political thought education, we can start from the following aspects: ① renew the learning concept; ② establish the concept of active learning; ③ strengthen the participation of the main body and promoting the development of online teaching; and ④ strengthen the technical training of students and improve the application ability of network teaching. Under the premise that society and schools have invested in the construction of network resources, the students' time and energy in using network resources are too low, which is bound to reduce the effectiveness of using network resources in teaching. Therefore, it is necessary to enhance the network awareness of teachers and students. Through strengthening education, students can fully realize the importance and richness of network information, and enhance their awareness of actively using network resources. The learning effect of students is closely related to the content of resources provided by teachers to students. When students are confused about some political information and ideological connotations in the process of self-study, they must be able to receive available information from the network materials provided by the schools, and cultivate students to form a good habit of viewing network resources. However, it should be noted that no matter how advanced the educational technology is, it also serves educational thought and educational goal. It is not allowed to put the cart before the horse, blindly pursue the advanced network technology and ignore the teaching rules and objectives, and turn the political thought teaching course into a demonstration course of technical operation. In the process of establishing and perfecting the cooperative education mechanism of college students' political thought education, the cooperation of educational objects plays an important role in stimulating the enthusiasm of educational subjects, promoting the efficient operation of the mechanism, and improving the education level of political thought education.

Teaching subjects mainly include “teachers' group, students' group, teachers' individual, and students' individual,” and all subjects have a close relationship. Each teaching subject plays a different role in the network teaching process. Among them, teachers and students have the greatest influence on teaching. The standardization and demonstration of textbooks can neither be altered, nor can the leading role of teachers in instruction be diminished or ignored. A good audio-visual operator who is not also a good teacher will lose sight of the true goal of educational reform and may even fail to accomplish the objectives of the lesson plan. The teaching environment, which includes teachers' values and the overall social environment of education, is an external factor that directly influences how education is implemented and has an impact. College students' political thought education will be directly impacted by the teachers' personal and professional values. Text, audio, video, and other media are examples of the types of teaching resources available on campus. These resources are essentially presented as partitions within the campus network, allowing students to precisely find the information they are looking for using keywords. The use of information technology, particularly its vast resources, variety of forms, and other qualities, determines that contemporary information technology can be created into a student-centered and teacher-led learning environment, which can effectively improve course instruction while also enhancing students' independence, innovation in thinking and writing, and ability to pursue careers. The main components of network literacy are knowledge and skills for using the network; the capacity for dialectical thought to comprehend, analyze, and evaluate network information; the development of legal and ethical principles in network communication; and the behavior habit of using a healthy network. The majority of college students are accustomed to using the Internet to look up information because it has so many informational resources available. The teaching of political thought courses is a special teaching process, so if institutions of higher learning want to master the dominant position of public opinion, they must make sure that the resources in the campus network have viewable value. The organic unity of knowledge and skills, process and method, emotional attitude, and values is one of the teaching goals of a political thought course.

The article "Analysis of Network Resources Integration of Political Thought Courses in Institution of Higher Learning Based on Collaborative Education Environment" was retracted in 2023. Reasons: unreliable results or conclusions; concerns about the data; concerns about the results or conclusions; concerns about the peer review.

### 3.3. Construction of the Network Resource Integration Model of Political Thought Courses

Rich network teaching resources are a necessary prerequisite for carrying out network teaching successfully and enhancing its impact. We can take action to improve teachers' and students' awareness of network teaching resources and enrich those resources to improve the impact of network teaching in light of the current low utilization rate and insufficient content of network teaching resources. Based on the concept of collaborative education, this article analyses the integration of network resources for political thought courses in higher education institutions and develops a model for such integration. The goal of DM is to extract implicit knowledge and rules from a large collection of imperfect, noisy, fuzzily, or randomly generated data. These knowledge and rules reveal some useful information and contain the precise relationship between a collection of database objects. From a database perspective, we define data mining (DM) as the process of extracting useful and fascinating information from the data set kept in a data warehouse or database. Education-related data mining (EDM) is the process of turning unusable data from various educational systems into knowledge that can be used by educators, students, and their parents, as well as educational researchers and software developers. DM steps are shown in Figure 2.

The article "Analysis of Network Resources Integration of Political Thought Courses in Institution of Higher Learning Based on Collaborative Education Environment" was retracted in 2023. Reasons: unreliable results or conclusions; concerns about the data; concerns about the results or conclusions; concerns about the peer review.

In this article, there are two main components that make up the resource integration techniques. The first component is technical, and it consists of an Arduino device identification program based on convolution NN that enables the program to classify and identify Arduino devices. The second component consists of learning resources. The creation of the Arduino device learning resources database is finished by gathering and screening the current learning resources, then turning them into videos. Data from various data sources must be combined into one format in order to make mining easier. Currently, a variety of technologies can be used for data transformation, including aggregation, missing value processing, continuous column transformation into discrete columns, and data type transformation. The most popular partition clustering algorithm is K-means. The clustering algorithm K-means is used to separate and identify differences between data elements. It begins by choosing K initial clustering targets from the sample set, then computes the distances between the sample data objects in accordance with the requirements of the rule algorithm, examines how the sample data objects are grouped in light of the computation results, and obtains K clustering results through iterative calculation up until the clustering center remains constant. Until the criterion function converges, the K-means algorithm repeatedly allocates data objects and creates new cluster centers. The formula illustrates the criterion:

(1) $$\begin{array}{c} E=\sum_{i=1}^{k}\sum_{x\in C_{i}}{\left|x-{\bar{x}}_{i}\right|}^{2}, \end{array}$$

where *x* is the data object in the dataset cluster *C*_*i*_; ${\bar{x}}_{i}$ is the calculated mean of the cluster; and *E* is the sum of squared errors of all the data objects in the dataset. The criterion function aims to produce clusters that are as compact and independent as possible, meaning that there is little similarity between clusters and lots of similarity within clusters. The updated calculation method for the cluster center in the conventional K-means algorithm is changed as follows in this article:

(2) $$\begin{array}{c} z_{i}=\frac{1/n_{i}\sum_{j=1}^{n_{i}}x_{j}^{\left(w\right)}-z_{i-1}}{2}. \end{array}$$

The next step is to determine by formula whether the confidence of frequent itemsets meets the requirement of minimum confidence given that all frequent itemsets satisfy the minimum support requirement. Strong association rules are those itemsets that satisfy both minimum support and minimum confidence. The equation reads as follows:

(3) $$\begin{array}{c} \text{Confidence}\left(A\Rightarrow B\right)=\\ P\left(A\cup B\right)=\frac{\text{Support}\_\text{Count}\left(A\cup B\right)}{\text{Support}\_\text{Count}\left(A\right)}. \end{array}$$

The association rules are generated through the following steps: first, all non-empty subsets *s* of each frequent itemset are generated; for each non-empty subset *s*, if

(4) $$\begin{array}{c} \frac{\text{Support}\_\text{Count}\left(l\right)}{\text{Support}\_\text{Count}\left(s\right)}\geq \text{Minimum Confidence.} \end{array}$$

Then, the output rule is

(5) $$\begin{array}{c} s\Rightarrow \left(l-s\right). \end{array}$$

Cross entropy is a widely used loss function. This article also uses cross entropy as the loss function. The formula of cross entropy is

(6) $$\begin{array}{c} H\left(p,q\right)=-\sum_{x}p\left(x\right)\log\;q\left(x\right). \end{array}$$

When it is used as the loss function of NN, *p* represents the correct answer and *q* represents the predicted value. The smaller the cross entropy is, the closer the two probability distributions are, which means that the constructed NN model is better.

The article "Analysis of Network Resources Integration of Political Thought Courses in Institution of Higher Learning Based on Collaborative Education Environment" was retracted in 2023. Reasons: unreliable results or conclusions; concerns about the data; concerns about the results or conclusions; concerns about the peer review.

In order to judge whether the iterative process is over or not, this article follows the construction idea of K-means algorithm criterion function, and defines a criterion function with the following formula:

(7) $$\begin{array}{c} E=\sum_{h=1}^{k}\sum_{x\in c_{h}}{\left|w-s\left(c_{hc},x\right)\right|}^{2}. \end{array}$$

Among them, *k* is the number of clusters into which the dataset is divided; *w* is the dimension of the data objects in the dataset; *x* represents the data objects in the cluster *c*_*h*_; and *c*_*hc*_ represents the cluster center of the cluster *c*_*h*_. That is, *s*(*c*_*hc*_, *x*) is the similarity between the data object and the cluster center. Suppose there are two data objects *x*, *y* with dimension *w*; the similarity measure is defined as

(8) $$\begin{array}{c} s\left(x,y\right)=\sum_{m=1}^{m=w}f\left(x_{m},y_{m}\right). \end{array}$$

Among them,

(9) $$\begin{array}{c} f\left(x_{m},y_{m}\right)=\left\{\begin{array}{cc} 1, & x_{m}=y_{m},\\ 0, & x_{m}\neq y_{m}. \end{array}\right. \end{array}$$

Based on the executed DM task, this step is to apply the algorithm to the transformed data to generate the desired mining results. This includes two stages: model construction and model evaluation. Mining association rules from the data in the training sample set database to guide the correction of evaluation index weights. In the process of training and testing, in order to provide the basis for later data analysis, effective rules can be stored in the rule base. Set by the log administrator. By extracting the access log, we can get all kinds of users' behaviors on the site, and it has a good effect on static pages. The background database records the registration information and online submission information of users. Through the method provided by the dynamic web technology, the access information of the client can be provided and the information extracted by the user can be collected. How to submit the results of DM to users is critical, because the usefulness of DM results mainly depends on this step. In the last step of knowledge discovery, various visualization tools and graphical user interfaces are usually used to show the results. In the part of index system revision, after training and testing the data of the training sample set database, the corresponding guidance information is obtained, and the weights of the evaluation indexes in the index database are adjusted, added, deleted, and modified.

The article "Analysis of Network Resources Integration of Political Thought Courses in Institution of Higher Learning Based on Collaborative Education Environment" was retracted in 2023. Reasons: unreliable results or conclusions; concerns about the data; concerns about the results or conclusions; concerns about the peer review.

## 4. Result Analysis and Discussion

The hardware setup for this experiment includes a 1 TB hard drive, a 2.13 GHz CPU, and 8 G of memory. The Windows operating system is used in the software environment. Using MatLab, we simulated the algorithm during the experiment and contrasted it with other algorithms. First, the values of other parameters, such as the basic learning rate and batch size, are fixed during the experiment in order to investigate the impact of iteration times on the model.  Table 1 displays the change in model accuracy over various iterations. In this study, data with iterations between 1000 and 12000 are chosen through analysis, and changes in the model's accuracy are noted.

Analysis of the data in the table shows that when the iterative operation of the model is short, the model does not learn enough about the features of the input image, the accuracy rate is not high, and the fluctuation of the accuracy rate is obvious. With the increasing number of iterations, the optimization algorithm of the network is constantly working, the network parameters are continuously optimized, and the test accuracy of the trained model is constantly improving.

Data cleaning, data integration, data transformation, and data reduction are the four steps that makeup data preprocessing. The purpose of data cleaning is to remove abnormal values and fill in any gaps in data. Data transformation is the process of transforming data into an analysis model for mining algorithms. Data integration is the integration of various data sources with the least amount of redundancy. To reduce the volume of mined data, use data reduction. We obtain the outcomes following mining and processing. From a variety of tree diagrams, we pick one representative tree area to examine and explain. A tree-like distribution diagram with three levels of nodes—each of which is the dimension referred to by the analysis result—represents the mining result.  Figure 3 depicts the clustering scenario when the data set contains less noise.  Figure 4 depicts the clustering scenario in a data set with a lot of noise.

The article "Analysis of Network Resources Integration of Political Thought Courses in Institution of Higher Learning Based on Collaborative Education Environment" was retracted in 2023. Reasons: unreliable results or conclusions; concerns about the data; concerns about the results or conclusions; concerns about the peer review.

As can be seen, the iterations of the two algorithms are roughly equivalent when there are not many isolated points and noise points. But when there are lots of isolated points and noise points, the cluster's center starts to stray from the actual cluster center. Additionally, this algorithm's convergence speed is unquestionably faster than other algorithms' when isolated points and noise points increase. The amplitude of each parameter update when training a NN is controlled by the basic learning rate. During the experiment, the values of other parameters, such as the number of iterations and the number of batch images, are fixed in order to investigate the impact of the basic learning rate on the model. The model accuracy for various rates of fundamental learning is shown in Figure 5.

By analyzing the data in Figure 5, we can find that when the learning rate is too small, the accuracy of the model is low and unstable. However, when the learning rate is high, the network parameters always move back and forth on both sides of the possible optimal value, and cannot converge to the optimal value. After analysis, the basic learning rate is set to 0.01.

If clustering and association rules mining are to be carried out, the original data collected must have a certain scale to ensure the rationality and effectiveness of the discovered rules, and the preprocessed data will eventually flow into the training sample set database. If the data are used for the evaluation of online learning, the amount of data is not allowed, and the result information obtained by analyzing the data flows into the training sample set database and the evaluation result database at the same time. With the continuous expansion of the database of training sample sets, the rules extracted by the system will become more scientific and reasonable. The recall rates of different algorithms are compared as shown in Figure 6. The accuracy comparison of different algorithms is shown in Figure 7.

Under different nodes of the allocation index tree, the cases and probability percentages of various types of resources will change, which indicates that the allocation status of resources is related to the visit volume and allocation index of the online course, and it also reflects that different types of resources have different influences on the visit volume and allocation index of the course. Batch number of pictures refers to that in the process of training, at the beginning of each iteration, a part of training data is selected first, and this part of data is the number of pictures processed by the network model in one iteration.  Table 2 shows the change in model accuracy when different batch pictures are set.

The article "Analysis of Network Resources Integration of Political Thought Courses in Institution of Higher Learning Based on Collaborative Education Environment" was retracted in 2023. Reasons: unreliable results or conclusions; concerns about the data; concerns about the results or conclusions; concerns about the peer review.

It can be seen that with the increasing number of batch images, the accuracy rate will be continuously improved within a certain number of images. However, when the number of batch images exceeds a threshold, the influence of the value of the batch images on the accuracy will decrease, and the accuracy of the model tends to be stable.

## 5. Conclusions

The majority of political thought instruction makes extensive use of network resources both during instruction and after class. By integrating political thought network resources with DM technology, knowledge acquisition processes can more effectively mine and analyze a sizable number of network teaching resources. This article carefully discusses and analyses the integration of network resources of political thought courses in institutions of higher learning from the perspective of collaborative education. In this article, the term “network resources” refers to all information sources that can be accessed online for use in the classroom when teaching political thought courses in higher education institutions. Additionally, a preliminary analysis of the key attributes of network resources is performed. Additionally, the design of an integration method for teaching resources is based on the idea of collaborative learning. This method includes the development of an Arduino device identification program based on NN and an Arduino device learning resource database. The study's findings demonstrate that the proposed algorithm is 95.11 percent accurate. The recall rate of this algorithm can reach 93.94 percent at the same time. By strengthening the development of network teaching subjects, enhancing network teaching resources, establishing a solid network teaching platform, and establishing a scientific operation evaluation mechanism, this article seeks to realize the cooperative education of political thought education and traditional education. The incorporation of online learning and courses into online teaching is influenced by a variety of factors. Our long-term research objective is to understand how to responsibly use DM technology, broadly uncover the correlation between various factors, and unearth insightful information for online instruction.

The article "Analysis of Network Resources Integration of Political Thought Courses in Institution of Higher Learning Based on Collaborative Education Environment" was retracted in 2023. Reasons: unreliable results or conclusions; concerns about the data; concerns about the results or conclusions; concerns about the peer review.

## Figures and Tables

**Figure 1:** Types of network teaching resources for political thought theory courses in institutions of higher learning.

**Figure 2:** DM steps.

**Figure 3:** Clustering when there is less noise in the dataset.

**Figure 4:** Clustering when there is a lot of noise in the dataset.

**Figure 5:** Model accuracy of different basic learning rates.

**Figure 6:** Comparison of recall rates of different algorithms.

**Figure 7:** Comparison of accuracy of different algorithms.

**Table 1:** Accuracy of models with different iteration times.

Iterations	1000	3000	6000
Accuracy rate	20%–50%	35%–70%	65%–80%
Iterations	8000	10000	12000
Accuracy rate	35%–55%	30%–90%	35%–35%

**Table 2:** Model accuracy of different batch pictures.

Batch number of pictures	15	30	50
Accuracy rate	56.31%	76.84%	86.67%
Batch number of pictures	80	120	160
Accuracy rate	86.31%	90.34%	92.35%

## Data Availability

The data used to support the findings of this study are available from the author upon request.
